# DSM and Optimization of Multihop Smart Grid Based on Genetic Algorithm

**DOI:** 10.1155/2022/5354326

**Published:** 2022-06-10

**Authors:** Qi Zhu, Yingliang Li, Jiuxu Song

**Affiliations:** School of Electronic Engineering, Xi'an Shiyou University, Xi'an 710065, China

## Abstract

Multihop smart grid is built on the basis of an integrated and high-speed communication network. Through the application of advanced sensing and measurement technology, equipment technology, control method, and advanced decision support system technology, the goal of reliable, safe, economic, efficient, environment-friendly, and safe use of the power grid is realized. In order to solve the problem of excessive demand for power supply, new energy power generation and demand response are proposed. According to the above background, the demand side economic scheduling problem is a complex optimization problem, which is difficult to be solved by ordinary algorithms. The adaptive global search algorithm based on a genetic algorithm can better solve complex optimization problems. The genetic algorithm proposed in this paper can effectively manage a large number of controllable loads in the selected area. The algorithm minimizes the cost and peak to the average ratio by changing the load. Home users can arrange their maximum load when the price is low. The peak load of residential buildings decreased from 98.5 kw/h to 90 kw/h, and the peak load decreased by about 7.53%. Through appropriate load dispatching, users minimize the daily electricity charge, which is reduced from 1352 yuan to 1245 yuan per day, and the daily electricity charge is reduced by about 7.25%. In addition, the advanced measurement, communication, and control means under the framework of the smart grid also play a key role in promoting all aspects of demand side management (DSM).

## 1. Introduction

Smart grid technology in intelligent buildings is a technology that uses two-way transmission of information and power. Then, it creates an advanced energy transmission network, which has the characteristics of automation and distribution. Multihop smart grid is built on the basis of an integrated and high-speed communication network. Through the application of advanced sensing and measurement technology, equipment technology, control method, and advanced decision support system technology, the goal of reliable, safe, economic, efficient, environment-friendly, and safe use of the power grid is realized [1, 2]. In order to solve the problem of excessive demand for power supply, new energy power generation and demand response are proposed. In order to improve household energy efficiency, demand side intelligent power dispatching has become a hot topic in the research of multihop smart grids. DSM plays the role of a control unit in the smart grid. It is a process used to balance the energy demand and supply between users and energy providers [3, 4]. This balance is achieved by combining energy management and reliable communication. The purpose of this is to establish a real-time and effective connection between users and energy suppliers. On the premise of maintaining the comprehensive service level of electric energy, adopt reasonable distribution and regulation methods to reduce the total consumption and load level of electric energy so as to achieve the purpose of reasonable distribution of electric energy, improving load curve, improving power supply efficiency and level, and promoting the coordinated development of sustainable economy, energy, environment, and other factors. In the current research, in order to improve the system performance of wireless communication networks in a multihop smart grid system and make it more reliable and safe, a variety of wireless multihop network architectures have been applied to the multihop smart grid [5].

According to the above background, the demand-side economic scheduling problem is a complex optimization problem that is difficult to be solved by ordinary algorithms. The adaptive global search algorithm based on the genetic algorithm in this paper can better solve complex optimization problems. Then, the genetic algorithm is used to select the most discriminating features and reduce the computational complexity [6]. This algorithm can not only detect more discriminating features and save computing time but also improve the classification accuracy of the classifier to some extent [7]. The purpose of the genetic algorithm is to make the final load curve as close as possible to the target load curve and realize the goal of the DSM strategy [8, 9]. If the goal of DSM is to reduce the electricity bill, the target load curve will be the price of electricity in the electricity market. A genetic algorithm provides an approximately optimal solution to a given problem, and it has the potential to solve such complex problems. Therefore, this paper uses a genetic algorithm to improve the scheduling algorithm to solve the cost optimization problem.

Combined with the DSM in the smart grid system and the rate optimization of wireless multihop network in the smart grid system, it brings benefits to users and further improves the performance of the whole network. DSM strategy includes DSM controller, which is used to calculate the user side energy-saving control method of smart grid based on genetic algorithm. User side intelligent controller is used to disconnect or connect different types of loads [10]. The DSM controller takes the target load curve as the input and calculates the load to be transferred to meet the target load consumption [11]. The algorithm is flexible and completely independent of the standard used to generate the target load curve. Comprehensively monitor the power load of users, advocate the use of smart appliances and vigorously develop energy storage equipment, and encourage the generation of distributed green energy to go online. In addition, the advanced measurement, communication, and control means under the framework of the smart grid also play a key role in promoting all aspects of DSM. In this paper, I put forward the following innovations. The specific contents are as follows:

1. This paper constructs a multihop smart grid structure model. As the DSM structure model of multihop smart grid is based on a genetic algorithm, it is necessary to monitor and analyze a set of key indicators to reflect the credit situation of power customers. Therefore, it is an important link to establish a scientific credit evaluation index of power customers.
2. In this paper, the DSM system in the smart grid is constructed. In this paper, a multihop smart grid DSM system is constructed based on a genetic algorithm. The goal of DSM can maximize the use of renewable energy resources, improve economic benefits, and reduce the use of electric energy from the main distribution network, that is, reduce peak load demand.

The overall structure of this paper consists of five parts.

The first chapter introduces the background and significance of DSM in multihop smart grids. The second chapter mainly describes the related work of DSM in multihop smart grids at home and abroad. Chapter 3 constructs the DSM system model of the smart grid. The fourth chapter carries out the experiment and analyzes the results. The fifth chapter is a summary of the full text.

## 2. Related Work of DSM in Multihop Smart Grid at Home and Abroad

Chen et al. put forward that the demand side should be considered as the classification of consumer electrical appliances. In order to get a more perfect electricity consumption model, consider adding a distributed generation model on the demand side, in which the distributed generation model can supply part of users' demand through independent power generation and make better use of resources [12]. Yao et al. put forward the interruptible load model of demand side appliances, which can dispatch household appliances better and increase the elasticity of the demand side [13]. Arun and Selvan designed a scheduling framework for residential energy consumption in a real-time pricing environment. This framework tries to achieve an ideal trade-off between minimizing the electricity cost and minimizing the waiting time for each household appliance to run, and the ultimate goal is to reduce the electricity cost and peak-to-average ratio [14]. Liang et al. put forward that the main purpose of DSM technology is to reduce the peak load demand and operating cost of the system. Although power companies can provide incentives to their customers and indirectly control the load through customer load grouping, most of the methods used do not consider independent criteria and objectives [15]. Zhu et al. proposed a traffic scheduling algorithm based on instrument data acquisition in building LAN. This method can effectively avoid interference between data communication devices, realize efficient traffic scheduling and data transmission, and finally meet the requirements of smart grid applications [16]. Wang et al. developed a realistic model to calculate the price of smart grid in order to reduce users' expenses, in which a convergent distributed algorithm was introduced and an estimate of production cost was provided according to actual demand changes [17]. Jabash and Jasper considered the access of distributed generation model but did not classify household appliances and only uniformly dispatch household appliances. After the addition of distributed generation, there may be residual power after meeting the needs of users, so the access of the municipal power model is considered [18]. Xu et al. proposed to consider the access of municipal power model and distributed model and the classification of household appliances, which reduced the power consumption cost of users but did not consider the user comfort, and there will be new power consumption peaks and valleys [19]. Fernandez et al. proposed and studied a DSM system based on real-time information and proposed a centralized scheme and game theory method to reduce the power generation cost and peak-to-average ratio of the smart grid [20]. Scarabaggio et al. proposed that in smart grid, DSM strategy needs to deal with a large number of various types of controllable loads. In addition, the load can last for several hours. Therefore, the strategy should be able to handle all possible control of various controllable load durations [21].

This paper mainly studies the problems of DSM and rate optimization under information transmission in multihop smart grid systems. In this paper, the DSM of multihop smart grid is studied based on a genetic algorithm. This strategy is based on load transfer technology and can handle a large number of various types of equipment. The design and analysis of a multihop smart grid need basic insight into the influence of grid topology and big data integrated network control, as well as the complex interaction between physical layer and network layer, including supporting communication, information, network, and computing system. DSM emphasizes obtaining direct economic benefits on the basis of improving the efficiency of electricity consumption. It is an operational activity, which not only seeks efficiency but also pursues efficiency. In the operation process of electric power companies, on the premise of obtaining the permitted power-saving income, it is necessary to adopt the market means of encouragement to promote users to actively save energy and electricity. The simulation research is carried out on the user side of the smart grid in residential areas with various loads. The DSM strategy suitable for smart grids in the future is simply explained, the mathematical load transfer technology is formulated, the DSM strategy based on a genetic algorithm is put forward, and the simulation results are given. If large users have a large demand for electricity load, they can report it to the power grid company in advance. The power grid company can make preparations in advance, reasonably dispatch the power generation, respond to the peak load in time, reduce the reserve capacity of the whole power grid, increase the load rate of running generators, and improve the generator efficiency.

## 3. DSM System Model of Smart Grid

### 3.1. Proposal of Genetic Algorithm

As a classical optimization algorithm, a genetic algorithm is usually used to solve various optimization problems. Aiming at the optimization objective model in this paper, genetic algorithm mainly has the following four characteristics.

- Selection operation: select 90% of chromosomes through a roulette selection algorithm. Excellent individuals are retained, and poor individuals are also given some living space to avoid falling into local optimization.
- Crossover operation generates a random number and compares it with crossover probability. Cross operation shall be carried out if conditions are met.
- Mutation operation generates random numbers and compares the mutation probability. The mutation operation shall be carried out if the conditions are met.
- Elite selection operation sorts the fitness and selects 10% to insert into the population. In the iterative process, the number of chromosomes of the population is the same as that of the initial population.

The proposed DSM strategy realizes that the actual power consumption curve of each transfer device at the moment of connection is as close as possible to the target power consumption curve. A genetic algorithm describes a set of attributes as a specific pattern and returns it, which is the predicted value of the input features, and the output values can be discrete or continuous. The learning of discrete values is called classification, while a genetic algorithm makes decisions by performing a series of tests [22, 23]. Therefore, the input features selected by the genetic algorithm are used to classify different electrical appliances. Genetic algorithm advances and new populations are generated from contemporary populations through remains algorithm: single-point crossover and binary mutation. A large crossover rate ensures faster convergence of solutions, and a very large mutation rate may lead to loss of good solutions inherited from the previous generation and prevent premature convergence of algorithms. The main steps of the genetic algorithm are shown in Figure 1.

Peak cutting and valley filling technologies are mathematically expressed as follows:

(1) $$\begin{array}{c} \sum_{t=1}^{N}\left(P_{L}\left(kT\right)\right)-P_{o}{\left(kT\right)}^{2}, \end{array}$$

where *P*_*o*_(*kT*) is the target consumption curve of *kT* under time; *P*_*L*_(*kT*) is the actual consumption curve of *kT* under time.

This minimization problem is subject to the following limitations:

(2) $$\begin{array}{c} X_{nikT}>0. \end{array}$$

The number of devices transferred in a one-time step cannot be greater than the number of devices controllable in the current time step.

(3) $$\begin{array}{c} \sum_{kT=1}^{N}X_{nikT}>\text{Ctrlable}\left(i\right), \end{array}$$

where Ctrlable(*i*) is the controllable number of *n* type equipment in time step *i*.

The characteristics of demand-side management problems, for example, the connection time of equipment can only be delayed but not advanced, which can be expressed as follows:

(4) $$\begin{array}{c} X_{nikT}=0. \end{array}$$

Options specify the maximum allowable delay time of all devices and the number of possible time steps to which devices can be transferred.

After the completion of the genetic algorithm, the calculation results are reflected on each planning line in the form of pheromone, which is a part of the initial pheromone strength of the genetic algorithm. The other part is the pheromone constant given by the genetic algorithm according to the specific scale of the problem. These two parts are the initial pheromone of the genetic algorithm. Then, the pheromone update model updates the pheromone intensity. Under the smart grid based on a genetic algorithm, a more comprehensive and reasonable TOU price policy will be implemented, which can promote energy conservation and consumption reduction. Comprehensively implement the real-time electricity price system in all power consumption fields and inform power users of the electricity price in time so that users can choose their own power consumption mode according to their own needs and combined with the actual electricity price, so as to realize users' active load regulation and peak shifting and valley filling [24].

### 3.2. Demand Side Management System Model of Smart Grid

As the structural model of the multihop smart grid DSM system is based on a genetic algorithm, it is necessary to monitor and analyze a group of key indicators to reflect the credit situation of power customers. Therefore, the establishment of scientific power customer credit evaluation indicators is an important link in the establishment of the customer credit evaluation model [25, 26]. Through the benefit analysis of the example, it is found that under the premise of reasonable DSM, there will be better economic benefits and environmental protection benefits for power generation enterprises, power users, power grid enterprises, and the whole society. Scientific and reasonable real-time electricity price systems and information give users a great right of choice. Users can choose an efficient power consumption mode according to their own needs, actively mobilize users to participate in power distribution and dispatching, and realize the function of load peak shifting and valley filling. The composition of the current peak and valley electricity price and the change of the daily service cost policy cannot accurately reflect the current peak and valley electricity price. It is suggested to promote a flexible electricity price policy reflecting the power supply and consumption cost in different time periods. According to the actual statistical data of the customer service center of the power supply bureau, based on a large number of analysis and research, this paper constructs the power customer credit evaluation index system according to the following principles.

- Guiding principle.
- In order to evaluate the credit of electric power customers, it is necessary to select the change of index characteristics to be ahead of time so as to sensitively reflect the problems existing in the credit of electric power customers and the development trend of the problems.
- Principle of completeness.
- When analyzing the reasons why power customers do not pay the electricity bill, we should collect information such as the background, development process, and consequences of the phenomenon of nonpayment of electricity bills as comprehensively and systematically as possible.
- Principle of proximate cause.
- The index design is determined according to the nature and characteristics of the reasons that lead to electricity customers not paying electricity bills on time. Different reasons for electricity customers not paying electricity bills have different properties and characteristics.
- The principle of combining qualitative and quantitative analysis.
- In the credit evaluation of electric power customers, adopting different evaluation indexes according to the characteristics of different evaluation contents can more accurately reflect the current situation and trend of electric power customers' credit. The goal of the genetic algorithm in this paper is to maximize the classification performance and minimize the number of features. The individual is the binary sequence of extracted feature vectors, and its size is equal to the dimension of features. The structural model diagram of the multihop smart grid DSM system based on genetic algorithm described in this paper is shown in Figure 2.

The output power of the generator set is affected by wind speed, and the approximate expression of the relationship between power and wind speed is as follows:

(5) $$\begin{array}{c} p_{WV}^{t}\left(v\right)=P_{n}\frac{v^{t}-v_{i}}{v_{r}-v_{i}},v_{i}<v^{t}<v_{r}, \end{array}$$

where *P*_*WV*_^*T*^ is the output power of the system at *t*; *v*_*i*_ is the cut in and cut out wind speed; *v*^*t*^ is the actual wind speed at *t* time; *v*_*r*_ is the rated wind speed; *P*_*n*_ is the rated power.

Power generation is determined by the current light, external temperature, and temperature coefficient

(6) $$\begin{array}{c} P_{PV}^{t}=P_{stc}\frac{G^{t}}{G_{stc}}, \end{array}$$

where *P*_*PV*_^*t*^ is the output power of the system at *t* time; *G*^*t*^ is the light intensity at *t* time; *P*_*stc*_¸*G*_*stc*_ is the active power and light intensity under standard test conditions.

The traditional nonintrusive electrical monitoring method uses Fisher discriminant analysis to select features, and its objective function is as follows:

(7) $$\begin{array}{c} J={\left(\mu_{1}-\mu_{2}\right)}^{2}⊗\frac{1}{\sigma_{1}^{2}+\sigma_{2}^{2}}, \end{array}$$

where *J*=[*J*_1_, *J*_2_,……,*J*_*L*_]^*T*^, *L* are the total number of parameters; *μ*_1_, *μ*_2_, *σ*_1_, *σ*_2_ is the mean and variance of two different eigenvectors, respectively; ⊗ represents Hadamard product.

Active power *P*

(8) $$\begin{array}{c} P=\frac{1}{T}\int_{0}^{T}ui\;dt=\sum_{i=1}^{\infty }V_{i}I_{i}\cos\;\theta_{i}, \end{array}$$

where *V* is the voltage; *I* is current; *θ* is the included angle; The subscript *i* is the *i* dimensional component of voltage or current.

Reactive power *Q*

(9) $$\begin{array}{c} Q=\sum_{i=1}^{\infty }V_{i}I_{i}\sin\;\theta_{i}. \end{array}$$

Power factor angle *θ*

(10) $$\begin{array}{c} \theta =\text{arctg}\left(\frac{P}{Q}\right). \end{array}$$

Current distortion rate ITHD

(11) $$\begin{array}{c} \text{ITHD}=\frac{1}{I_{l}\sqrt{\sum_{i=2}^{\infty }I_{h}^{2}}}, \end{array}$$

where *I*_*l*_ is the fundamental current; *I*_*h*_ is the ratio of total harmonic current effective value to fundamental current.

It can be transferred to an appropriate time step by a genetic algorithm according to its importance. From the analysis of the results obtained from the genetic algorithm, it can be known that after DSM, the daily maximum load can be reduced, the daily minimum load can be increased, and the peak-valley difference can be reduced, which can play a role in shifting the peak and filling the valley. After selecting the individual with the highest fitness, it can carry out gene crossover and mutation operations on the population. Establish the cost compensation mechanism and incentive mechanism of DSM. Research and establish new energy demand side special management funds suitable for the development of smart grid, make up for the cost of power grid enterprises to carry out power DSM, strive to break the power grid enterprises' pursuit of power sales interests, reform the assessment system, and increase incentives for power grid enterprises to take the leading force to deeply carry out power DSM.

### 3.3. Constructing DSM System in Smart Grid

DSM includes technologies and policies aimed at balancing daily energy consumption. Compared with the management scheme of adding new generator sets and other power suppliers, DSM is not only to increase the supplied energy but also to control the consumption form by using energy management technology. The most important goal of DSM is to reduce the peak value. In this paper, a multihop smart grid DSM system is constructed based on a genetic algorithm. The goal of DSM can maximize the use of renewable energy resources, improve economic benefits, and reduce the use of electric energy from the main distribution network, that is, reduce peak load demand. Multihop smart grid managers design the target load curve through the target of DSM system. Smart grid provides two-way interactive marketing technology and mechanism support, which makes the implementation of DSM naturally transition from the past government behavior and policy orientation to the market mechanism. In the past, due to the lack of advanced measurement and communication means, it was impossible to give convincing information on income sharing and investment return of DSM measures, which was effectively solved in the smart grid era. The front-end management software of DSM can realize remote power consumption information data collection and remote power distribution fault diagnosis according to user requirements.

The common technologies of DSM in smart grids are as follows.

- Increase nonpeak load
- When the production cost in off-peak hours is lower than that in peak hours, this promotes energy consumption in off-peak hours. Various incentives, such as discounts, can encourage consumers to change their consumption habits.
- Strategic power saving
- Strategic power saving mainly reduces the periodic consumption of energy by reducing the waste of energy so as to improve the efficiency of energy consumption. The program includes a variety of incentives, mainly for technological change.
- Strategic load growth
- Strategic load growth increases periodic energy consumption. Power suppliers achieve this goal by deploying intelligent systems, node equipment, and more competitive energy.
- Elastic modeling
- This strategy is more flexible and needs modeling to be carried out according to the needs of consumers at every moment. By installing load-limiting devices, this strategy will limit consumers' energy use for certain periods of time without affecting the actual and safety conditions.

The software system supports various channel modes, Chinese information, centralized and remote reading of electricity consumption information of multifunction meters, parameter setting and correction, data sharing of demand-side user terminals, real-time copying of abnormal data analysis of terminals, fault event information recording, etc. DSM system emphasizes the establishment of a partnership between power companies and users. It is required to establish a very harmonious cooperative feeling between power companies and users so as to share risks and gain benefits for the benefit of power supply and electricity consumption. The system can also automatically analyze and judge the historical operation data of power users and remind the power demand side operation management personnel to make relevant inspections by voice, curve, report form, etc, for users who may steal electricity and leak electricity, so as to improve the efficiency of power supply reliability analysis of distribution branches and on-site power dispute handling by operators.

## 4. Experimental Results and Analysis

### 4.1. Experimental Analysis

The genetic algorithm is applied to the power demand dispatching management of a residential building in a community of a city. The building has more than 1000 controllable basic household appliances with different rated power in 6 different types. Generally speaking, the residential load has the characteristics of low power consumption and small duty cycle. Different types of household appliances and their rated power are shown in Table 1.

It can be seen from Table 1 that among different types of household appliances, water heaters account for the highest energy consumption, followed by air conditioners, microwave ovens, computers, televisions, and finally, electric fans. Therefore, adopting reasonable optimization methods and adjusting the basic functions and structure of China's power, demand side can greatly improve the power supply and distribution capacity of the power grid, achieve energy conservation and consumption reduction, and promote the construction of a smart grid.

The load curve after load reduction by the genetic algorithm is shown in Figure 3.

As can be seen from Figure 3, the shape of the daily load curve has been obviously improved after the load is reduced by the genetic algorithm. From 20:30 to 22:30, the unplanned load was obviously reduced from 285 MW to 273 MW, effectively reducing the peak-valley difference, achieving the effect of demand-side management and improving the economy of power system operation.

After the real-time sales price is implemented, the daily maximum load appears at 20:30, and it is assumed that the maximum load that intelligent equipment can cut at each moment is predicted, as shown in Figure 4.

As can be seen from Figure 4, 7:00 a.m. to 9:00 a.m. and 17:00 p.m. to 19:00 p.m. are the peak periods of people's travel, and electric vehicles are in use, so the standby capacity is small. From 11:00 to 13:00 noon, a small number of car owners will go home for dinner, and the standby capacity is slightly reduced compared with working hours. At night, because the electric vehicle has been running during the day, the remaining power is not much, so the standby capacity will be much less than the working hours.

Calculate the load index of the active load curve before and after the adjustment of the real-time sales price model, as shown in Table 2.

It can be seen from Table 2 that after users adjust the load according to the real-time sales price, the load curve has changed significantly, the maximum load decreases, the minimum load increases, the peak-valley difference decreases, and the effect of shifting peak and filling valley is obvious, and the load tends to be stable, which can guide users to use electricity reasonably and optimize resource allocation.

Assume the relationship function between the compensation price and the load reduction of intelligent equipment, and the intelligent parameters of each node are shown in Table 3.

As can be seen from Table 3, the intelligent equipment compensation electricity price model program is called at 20:30, 21:00, and 21:30, respectively, [qzi, qz] = Zhen (30, 21, 0.5, [0120.80.900.60.600.60.80100) *P* > [01.9400.5520.9706.02002.3401.88000.55001.22000. 5500.7600.8800.8677058555. Actively promote the establishment of a new mechanism for unified planning, unified approval, and coordinated development of smart grid and distributed energy, as well as the market access mechanism, exit and stop operation boundary conditions of distributed energy, and promote the healthy and orderly development of distributed energy. Establish a scientific and reasonable electricity price system and form a comprehensive electricity price selected by users of the power supply according to the four periods of peak, peak, flat, and valley. According to the seasonal load requirements, some energy-saving and consumption-reducing electricity price incentives are formulated to reduce unnecessary power waste.

The running results of multihop smart grid scheduling using machine learning algorithm, ant colony algorithm, particle swarm optimization algorithm, and genetic algorithm in this paper are shown in Figures 5–7.

It can be seen from Figures 5–7 that the genetic algorithm proposed in this paper can effectively manage a large number of controllable loads in the selected area. The algorithm minimizes the cost and peak to the average ratio by changing the load. Home users can arrange their maximum load when the price is low. The peak load of residential buildings decreased from 98.5 kw/h to 90 kw/h, and the peak load decreased by about 7.53%. Through appropriate load dispatching, users minimize the daily electricity charge, which is reduced from 1352 yuan to 1245 yuan per day, and the daily electricity charge is reduced by about 7.25%.

### 4.2. Empirical Conclusion

The ultimate goal of DSM is to improve the power consumption efficiency of customers' power terminals. However, in the design process of DSM mode, users must actively participate and discuss the power supply mode and structure of DSM. In this paper, the genetic algorithm has been compared with other algorithms many times, and finally, it is concluded that the method in this paper is the most advantageous in the DSM of multihop smart grid. Because of the change of load type and capacity of the power demand side, the imperfect function of DSM technology, and other factors, it is difficult for power grid demand side dispatching to achieve the functions of supply and demand balance, energy saving, and safety, and there are some disadvantages such as increased power loss and high unit power production cost. From the analysis of the results obtained from the genetic algorithm, it can be known that after DSM, the daily maximum load can be reduced, the daily minimum load can be increased, and the peak-valley difference can be reduced, which can play a role in shifting the peak and filling the valley. It can also guide users to use electricity reasonably, optimize resource allocation, achieve the effect of energy saving, improve the economy and stability of power system operation, and finally achieve the purpose of DSM.

Based on a genetic algorithm, the real-time monitoring of power load is the basic guarantee for the construction of an intelligent DSM system. In the process of system construction, higher requirements are put forward for the metering system of power terminals. It is required that the metering system must have the function of real-time power load demand communication with the DSM system and obtain dynamic power grid parameters and load through the corresponding monitoring instruments. Using a genetic algorithm to carry out multiobjective optimization planning successfully solves the multiobjective, nonlinear, and discrete optimization problems in power grid planning and can simultaneously generate several optimization planning schemes in which each objective can be realized in different degrees, thus coordinating the conflicts among objectives and obtaining satisfactory results, which shows that this method is feasible.

## 5. Conclusions

The construction of an electric power company not only involves the huge economic benefits of users but also involves the economic development of the electric power system. This paper focuses on the application of multihop smart grid DSM based on a genetic algorithm. In the integrated model of DSM in this paper, through the genetic algorithm, firstly, the load response technology is established to dynamically adjust the load demand through the adjustment and change of real-time sales price. The smart grid has an advanced metering system and communication system, which provides conditions for load response technology. The control center can monitor the system operating parameters in real-time and transmit the real-time sales price to users. The genetic algorithm proposed in this paper can effectively manage a large number of controllable loads in the selected area. The algorithm minimizes the cost and peak to the average ratio by changing the load. Home users can arrange their maximum load when the price is low. The peak load of residential buildings decreased from 98.5 kw/h to 90 kw/h, and the peak load decreased by about 7.53%. Through appropriate load dispatching, users minimize the daily electricity charge, which is reduced from 1352 yuan to 1245 yuan per day, and the daily electricity charge is reduced by about 7.25%. The establishment of a reasonable management system, a scientific electricity price system, and an integrated monitoring system with a high level of automation through genetic algorithm can improve China's existing DSM system, achieve the purpose of peak load shifting and valley filling, energy conservation, and consumption reduction, and promote the construction of intelligent power demand side system and the sustainable development of power resources.

## Figures and Tables

**Figure 1:** Flow chart of genetic algorithm.

**Figure 2:** Structure model of multi-hop smart grid.

**Figure 3:** Load curve after genetic algorithm reduction.

**Figure 4:** Maximum load after genetic algorithm reduction.

**Figure 5:** Comparison of daily power consumption of residential buildings before and after planning.

**Figure 6:** Daily electricity consumption of residential buildings before and after planning.

**Figure 7:** Comparison of energy consumption of residential buildings before and after planning.

**Table 1:** Rated power of different types of household appliances in residential areas.

Equipment name	Energy consumption (kWh)	Quantity
Electric fan	0.07	135
Heater	4	136
Television	0.2	135
Microwave oven	2	135
Computer	0.6	67
Air conditioner	2.6	205

**Table 2:** Comparison of load indicators before and after real-time sales price model adjustment.

	Daily maximum load (MW)	Daily minimum load (MW)	Peak valley difference (MW)	Daily average load (MW)	Daily load rate (%)
Before adjustment	309.8948	244.3473	65.5471	277.2354	89.4612
After adjustment	301.2984	253.4577	47.8406	277.2347	92.0133

**Table 3:** Parameters of intelligent equipment.

Node number	Actual reduced load of chemical equipment			Default rate	Duration
	20:30	21:00	21:30		
1	1.931	1.942	1.961	0.35	2
2	0.551	0.553	0.571	0.26	2
3	0.972	0.971	0.992	0.21	0.7

## Data Availability

The dataset can be obtained from the corresponding author upon request.
